# Research on the Application of Intelligent Choreography for Musical Theater Based on Mixture Density Network Algorithm

This article has been retracted.

**DOI:** 10.1155/2021/4337398

**Published:** 2021-11-29

**Authors:** Jun Cang, Yichen Huang, Yanhong Huang

**Affiliations:** ^1^School of Economics and Management, Tongji University, Shanghai 200092, China; ^2^College of Music, Fujian Normal University, Fuzhou 350117, China

## Abstract

Musical choreography is usually completed by professional choreographers, which is very professional and time-consuming. In order to realize the intelligent choreography of musical, based on the mixed density network (MDN), this paper generates the dance matching with the target music through three steps: motion generation, motion screening, and feature matching. The choreography results in this paper have a high degree of matching with music, which makes it possible for the development of motion capture technology and artificial intelligence and computer automatic choreography based on music. In the process of motion generation, the average value of Gaussian model output by MDN is used as the bone position and the consistency of motion is measured according to the change rate of joint velocity in adjacent frames in the process of motion selection. Compared with the existing studies, the dance generated in this paper has improved in motion coherence and realism. In this paper, a multilevel music and action feature matching algorithm combining global feature matching and local feature matching is proposed. The algorithm improves the unity and coherence of music and action. The algorithm proposed in this paper improves the consistency and novelty of movement, the compatibility with music, and the controllability of dance characteristics. Therefore, the algorithm in this paper technically changes the way of artistic creation and provides the possibility for the development of motion capture technology and artificial intelligence.

## 1. Introduction

As a performing art form, dance is generally based on rhythmic movements to music. Choreography for musicals is usually done by talented professionals, which is challenging and time-consuming. Advances in technology are changing the way art is created, such as image style migration, handwriting generation, and other hot issues in computer vision research. The fusion of technology and art is the result of the use of computers to automate music-based choreography. When artists use technology as a way to create, this technology can serve as a catalyst of inspiration for artists and will bring great potential.

With the development and widespread application of motion capture technology, the realism of dance movements is guaranteed, but it is only a simple replication of data [1–3]. However, in many application areas such as games, animation, and virtual reality, there are interactive demands that require virtual characters to have creative human-like movements, such as dancing [4]. For the dance movements of virtual characters, especially the dance animations created manually by users, the animator needs to manually adjust the position and rotation of each bone of the model in key frames. Completing this task not only is very time-consuming but also requires the animator to be experienced, which greatly limits the development of virtual character dance animation. Therefore, a successful dance synthesis algorithm can be useful in areas such as music-assisted dance teaching [5–7], audio-visual game character movement generation [8, 9], human behavior research [10–13], and virtual reality.

This paper is divided into six parts: the first part introduces the background and research significance of musical intelligent choreography based on MDN. The second part introduces the research methods and research results in this field, as well as the research content and innovation of this paper. The third part introduces the model structure of the action generation model used in this paper, as well as the parameter selection in the process of model training and prediction. The fourth part puts forward the multi-level feature matching algorithm of music and action and arranges the dance actions generated in the third chapter according to the characteristics of the target music. The fifth part verifies the effectiveness of the musical intelligent choreography scheme based on MDN. The sixth chapter summarizes the current work and research results.

## 2. Related Work

At present, many scholars have conducted a lot of research on the problem of computer music choreography and obtained many valuable results. Zhong et al. proposed the rhythm analysis method, which defines the rhythm of the movement based on the changing speed of the vertical direction of the foot and the hand displacement and uses the extreme value point of the joint angular velocity as the rhythm segmentation point, whereby the movement characteristic curve is refitted [14]. Yang et al. obtained that the rhythm features were added to the intensity features, where the action intensity features were based on the concept of force in the Laban movement system and the music intensity features were defined based on audio energy and sound pressure [15]. Ofli et al. added transition frame interpolation and path control algorithms to the rhythm and intensity feature matching algorithm to make the dance movements more natural and enrich the spatiality of the dance [16]. In recent years, the development of deep learning techniques has provided methods for extracting high-dimensional features from raw data and has opened up new possibilities in the fields of motion generation and automatic music choreography [17–21]. Recurrent neural network (RNN) has been considered as an effective means to solve sequential tasks and has been used in natural language processing (NLP) [22], speech recognition [23], music composition [24], and other fields. However, traditional RNNs suffer from the gradient disappearance problem, which can seriously affect the effect when the sequence length increases. For this reason, Wei et al. proposed long short-term memory (LSTM). This network retains the basic model of RNN and replaces the normal nodes (usually tanh) in RNN with long short-term memory nodes to make it have the sequence processing capability of RNN while improving the gradient vanishing problem, so it is widely used in sequence data processing tasks [25–30].

In summary, although there is a certain amount of research on computerized automatic music choreography technology, it is not advanced enough. The existing research mainly has the following problems: the novelty and consistency of the generated movements need to be improved; the generated movements and the beat of the music need to be strengthened; the current research does not give much consideration to the user's human control of the choreography results.

Based on the above background, this paper proposes an automatic music choreography algorithm, which is based on a large amount of existing music and dance data, and uses a deep learning algorithm to train a model that can combine filtering conditions to automatically and intelligently generate dance movements that meet expectations and choreograph according to the matching of music and movement fragments. The algorithm can generate novel and creative dance movements and replace the traditional choreography algorithm, greatly improving efficiency and saving choreography cost, which has practical value.

### 2.1. Hybrid Density Network-Based Action Generation Algorithm

With the development of computer animation and robotics, more and more applications require a large amount of real human motion data, which cannot be satisfied by motion capture and manual production alone, so researchers have started to tackle the problem of motion generation. Broadly speaking, action generation algorithms can be divided into two categories: one for combining new action sequences by reusing and editing existing action fragments in the database, and the other for generating completely new action sequences by learning the mapping and constraint relationships within action data through neural networks. For automatic computer choreography tasks, the traditional dance synthesis algorithms based on matching music and movement features belong to the first category, where the synthesized dance movement sequences are derived from movement fragments in the database with limited dance diversity. In order to generate novel movement data, machine learning and deep learning algorithms have been applied in the field of movement generation [31–35]. Hidden Markov models (HMMs), Gaussian processes, and dimensionality reduction techniques can capture the intrinsic dependencies and potential correlations of movement data, but compared with the powerful learning ability of neural networks, traditional machine learning methods are restricted in their ability to capture data changes. Therefore, in this paper, we choose to use a deep learning-based sequence generation model for action generation.

In order to train a motion generation model, a motion dataset needs to be constructed and the motion data are represented in vector form as the input features of the model. Due to the limited number of publicly available motion capture datasets, with only a small fraction of dance movements and even fewer complete choreographic movements accompanied by music, the amount of data is not sufficient to accomplish the task of deep learning. Therefore, this paper constructs a dataset using motion files in Vocaloid Motion Data (VMD) format obtained from the web and trains a motion generation network with it.  Table 1 shows some of the data obtained by parsing the bone keyframe data blocks in the VMD file.

In order to implement an effective computer choreography algorithm to ensure that the choreographed dances are realistic and novel enough, rather than relying on user hand-crafted and motion-captured data, the motion generation problem needs to be solved. Therefore, this paper additionally constructs a music-motion dataset consisting of complete music choreography sequences. The music and dance styles contained in the dataset constructed in this paper are not exactly the same, and there are fast and slow speeds, so it is necessary to classify the actions before the network training.  Table 2 shows the number of frames and duration of various types of movements after classification, and Figure 1 shows the comparison of movements at different speeds.

In this paper, we construct an action generation model based on MDN, which consists of two parts, a neural network and a hybrid density model. Specifically for the task of this paper, the preceding neural network is an action prediction network, which predicts the action of the next frame based on the input of several frames of action data and the output of the network is used as a parameter vector to parameterize the hybrid density model later, so as to determine the mean, variance, and weight occupied by each hybrid component. The final output of the whole model is not a single skeletal position tensor, but the probability density of each dimension in the tensor. The overall model schematic is shown in Figure 1.

The action prediction network is a neural network used to learn the internal dependencies and mapping relationships between action sequence data. After parameterization of the model, the final output is the probability density *p*(*t|x*) of each parameter of the spatial location of each node in the next frame, which is given by the following equation:

(1) $$\begin{array}{c} p\left(t|x\right)=\sum_{i=1}^{m}\alpha_{i}\left(x\right)\varphi_{i}\left(t|x\right). \end{array}$$

In order to balance the effect and complexity of the model, the Gaussian kernel function is used, *φ*_*i*_(*t|x*), to represent each mixture component in the mixture density model, which is given by the following equation:

(2) $$\begin{array}{c} \varphi_{i}\left(t|x\right)=\frac{1}{{\left(2\pi \right)}^{c/2}\sigma_{i}{\left(x\right)}^{c}}e^{-\left({\left\|t-\mu_{i}\left(x\right)\right\|}^{2}/2\sigma_{i}{\left(x\right)}^{2}\right)}. \end{array}$$

Let *m* be the number of components in the mixture component and *c*=63 be the dimensionality of the LSTM output data; then, the output of the MDN is a tensor *z* containing the number of variables *m*(*c*+2), which includes all the parameters needed to construct the mixture model, with the following equation:

(3) $$\begin{array}{c} z=\left[z_{1}^{\alpha },\ldots ,z_{m}^{\alpha },z_{m+1}^{\mu },\ldots ,z_{mc+m+1}^{\mu },z_{mc+m+2}^{\sigma },\ldots ,z_{m\left(c+2\right)}^{\sigma }\right]. \end{array}$$

Using the parameter vector, the entire part of the mixed density model can be encoded as a simple error measure where the error function is a negative log-likelihood function (for the *q*-th sample).

(4) $$\begin{array}{c} E^{q}=-\log\left[\sum_{i=1}^{m}\alpha_{i}\left(x^{q}\right)\varphi_{i}\left(t^{q}|x^{q}\right)\right],\\ \alpha_{i}=\frac{e^{z\left(\alpha /i\right)}}{\sum_{j=1}^{M}e^{z\left(\alpha /j\right)}|}, \end{array}$$

where *σ*_*i*_=*e*^*z*_*i*_^*σ*^^, *μ*_*i*_=*z*_*ik*_^*μ*^,  and *α*_*i*_ is the mixing factor of each mixture component for input *x*.

The action generation model consists of three LSTM layers, three fully connected layers (dense) and a tandem operation (concatenate), and the specific network structure is shown in Figure 2.

The formula for calculating the gradient involved in the training process is as follows:

(5) $$\begin{array}{c} \frac{\partial E^{q}}{\partial z_{k}^{\alpha }}=\alpha_{k}-\frac{\alpha_{k}\varphi_{k}}{\sum_{j=1}^{m}\alpha_{j}\varphi_{j}},\\ \frac{\partial E^{q}}{\partial z_{ik}^{\mu }}=\frac{\alpha_{i}\varphi_{i}}{\sum_{j=1}^{m}\alpha_{j}\varphi_{j}}\frac{\mu_{ik}-t_{k}}{\sigma_{i}^{2}},\\ \frac{\partial E^{q}}{\partial z_{i}^{\sigma }}=-\frac{\alpha_{i}\varphi_{i}}{\sum_{j=1}^{m}\alpha_{j}\varphi_{j}}\left\{\frac{{\left\|t-\mu_{i}\right\|}^{2}}{\sigma_{i}^{2}}-c\right\}. \end{array}$$

To obtain good results in the training of deep neural networks, it is necessary to provide enough data so that the neural networks can fully explore the intrinsic relationships among the data. For training, a mixture model (*m*=12) with 12 Gaussian distributions is used, the number of LSTM nodes per layer is set to 512, the batch size is set to 100, the length of the sequence is set to 120, and the learning rate is set to 1 × 10^−3^, with a total of 500 training cycles, using the RMS Prop optimizer is used for optimization.

The model training process requires a minimization error function different from other loss functions commonly used in networks (such as cross entropy, etc.), where *E*^*q*^ does not satisfy the condition of the constant greater than zero, so when the model loss is less than zero, it will continue to decline with training, as shown in Figure 3.

The loss of the validation set and the loss of the training set are not in the same direction, and there is not even a significant downward trend. This is because the dance action generation task is different from other tasks such as target classification, and the choreography and expression of dance actions are not unique, which is where the diversity of dance actions lies, and the training process of the action generation model is to find regularity in them, as shown in Figure 4.

### 2.2. Choreography Based on Music and Movement Characteristics

#### 2.2.1. Analysis of the Overall Characteristics of Music

In this paper, a multilevel music and action feature matching algorithm is proposed. When performing computerized music choreography, the overall characteristics of the target music are first analyzed and initially matched with the action characteristics; after that, the degree of matching between the local characteristics of the music segments and the action fragments is considered and the action sequence matching with the target music is obtained according to the feature matching of the rhythm and intensity as well as the results of the connect ability analysis; finally, the adjacent action fragments of this action sequence are interpolated and connected to the final choreography result obtained, and the computerized automatic music choreography task is completed.

The input audio signal *x*(*n*) is transformed by CQT to obtain *X*(*n*, *k*) by the following equation:

(6) $$\begin{array}{c} X\left(k\right)=\frac{1}{N_{k}}\sum_{n=0}^{N_{k}-1}x\left(n\right)w_{N_{k}}\left(n\right)e^{-j\left(2\pi Q/N_{k}\right)}. \end{array}$$

Let *d*(*n*, *k*) denote the energy increment of the music signal from frame *n* − 1 to frame *n* at the frequency of *f*_*k*_, and the denoising process is performed as follows:

(7) $$\begin{array}{c} d\left(n,k\right)=\left\{\begin{array}{cc} \max & \left(X\left(n,k\right),X\left(n+1,k\right)\right)-\mathrm{PrePow}\left(n,k\right),\\ \min & \left(X\left(n,k\right),X\left(n+1,k\right)\right)\geq \mathrm{PrePow}\left(n,k\right),\\ 0 & \text{else}, \end{array}\right. \end{array}$$

where PrePow(*n*, *k*)=max(*X*(*n* − 1, *k*), *X*(*n* − 1, *k* − 1), *X*(*n* − 1, *k*+1)). The final spectral energy abrupt change point function value *D*(*n*), which is the sum of the increments of each frequency at the current moment, is as follows:

(8) $$\begin{array}{c} D\left(n\right)=\sum_{k}d\left(n,k\right). \end{array}$$

The next step is to estimate the beat period. Based on the periodicity of the beat, the beat period is predicted as AC(*τ*) by calculating the value of the autocorrelation function of the note onset:

(9) $$\begin{array}{c} \text{AC}\left(\tau \right)=\sum_{n=1}^{len/2}D\left(n\right)*D\left(n+\tau \right),\tau \in \left(0,\frac{\text{len}}{2}\right), \end{array}$$

where Len is the total length of the music sequence. The *τ*_max_ period of the estimated music beat is the one where AC(*τ*) takes the maximum value. Due to the periodicity of the music beat, it is known that there are more than one *τ*, where AC(*τ*) represents multiples of the *τ*_max_ maximum value. Thus, by averaging, we can obtain the beat length *τ*_max_. After obtaining the beat length, the corresponding beat per minute (BPM) is 60/*τ*_max_.

#### 2.2.2. The Overall Characteristics of the Music and the Action Matching

The action data used in this paper are sampled at a frequency of 30 frames/second, and the three-dimensional spatial coordinates of each joint point at the corresponding moment of each frame are recorded, so the distance between the positions of the corresponding joints in two adjacent frames can be approximated as the velocity of the joint at that moment and the average velocity *v*_*i*_^Arm^ of the arm of the action segment *N*_*i*_ is

(10) $$\begin{array}{c} v_{i}^{\text{Arm}}=\sum_{f=1}^{L_{\text{Motion}}^{-1}}\frac{\left\|p_{f+1}^{\text{Arm}}-p_{f}^{\text{Arm}}\right\|}{L_{\text{Motion}}-1}, \end{array}$$

where *f* is the number of dams in the *N*_*i*_ action clip, *L*_Motion_ is the length of the action clip, and *p*_*f*_^Arm^ represents the position of the arm joint in the first *f* frame. The arm joint in equation (10) can also be replaced by other joint positions to calculate the average velocity of other joints.

The spatiality measure *e*_*i*_ of the action fragment *N*_*i*_ is

(11) $$\begin{array}{c} e_{i}=\sum_{f=1}^{L_{\text{Motion}}-1}\frac{\sqrt{{\left(x_{f+1}^{\text{Root}}-x_{f}^{\text{Root}}\right)}^{2}+{\left(y_{f+1}^{\text{Root}}-y_{f}^{\text{Root}}\right)}^{2}}}{L_{\text{Motion}}-1}, \end{array}$$

where *x*_*f*_^Root^ and *y*_*f*_^Root^ are the *y* coordinates of *x* root nodes of the first *f* frame, respectively.

When the target music is input, the overall features, i.e., BPM and average duration of change notes, are first extracted, the most likely dance style and dance speed corresponding to the target music are judged, and the corresponding movement generation model is selected to generate movements.

### 2.3. Rhythm- and Intensity-Based Music and Movement Feature Matching

For the purpose of description, the whole target music is given as *M*, which is divided into *m* music pieces after music segmentation, i.e., *M*_1_, *M*_2_,…, *M*_*m*_:

(12) $$\begin{array}{c} M=\left[M_{1},M_{2},\ldots ,M_{m}\right]. \end{array}$$

The music features used for local feature matching in this paper consist of two parts: rhythm and intensity features. The features of the music fragment *M*_*i*_(1 ≤ *i* ≤ *m*) are

(13) $$\begin{array}{c} \text{music feature}\left(f\right)=\left[\begin{array}{c} F_{R}^{\text{Music}}\left(f\right)\\ F_{l}^{\text{Music}}\left(f\right) \end{array}\right],\;f\in M_{i}, \end{array}$$

where *f* is the frame number of the music clip and *F*_*R*_^Music^ and *F*_*l*_^Music^ are the rhythm and intensity characteristics of the music clip *M*_*i*_, respectively.

Assuming that the current beat position is *T*_*n*_, the next beat position can be predicted as

(14) $$\begin{array}{c} T_{n+1}^{\prime }=T_{n}+\tau_{\max}. \end{array}$$

In summary, the rhythmic characteristics of the music clip *M*_*i*_ are

(15) $$\begin{array}{c} F_{R}^{\text{Music}}\left(f\right)=\left\{\begin{array}{cc} 1, & f\text{ is the beat moment,}\\ 0, & \text{else,} \end{array}\right.\;f\in M_{i}. \end{array}$$

In order to calculate the intensity characteristics of the music, the CQT spectrum is obtained by CQT transformation of the music fragment. The average energy of the *k*th *M*_*i*_ semitone of the music fragment is

(16) $$\begin{array}{c} \bar{X}\left(k\right)=\frac{1}{\left|M_{i}\right|}\sum_{n\in M_{i}}X\left(n,k\right), \end{array}$$

where, |*M*_*i*_| is the total number of music segments *M*_*i*_ and *X*(*n*, *k*) represents the frequency amplitude of the *k*th semitone of the *n*th music signal. The local peak of the average energy is

(17) $$\begin{array}{c} X_{\text{peak}}\left(k\right)=\left\{\begin{array}{cc} \bar{X}\left(k\right), & \bar{X}\left(k\right)\geq \bar{X}\left(k\mp 1\right),\\ 0, & \text{else.} \end{array}\right. \end{array}$$

Considering the auditory characteristics of human ear and the amplitude and frequency of signal, the approximate sound pressure level is used as the characteristic of music intensity.

(18) $$\begin{array}{c} F_{I}^{\text{Music}}\left(f\right)=\;\log_{10}\left(\sum_{k=C4}^{C6}X_{\text{peak}}{\left(k\right)}^{2}\cdot f_{k}^{2}\right),\;f\in M_{i}, \end{array}$$

where *f*_*k*_ is the frequency value corresponding to the tone groups C4–C6.

Similar to the musical characteristics, the action characteristics in this section are also used for the action segments. The action sequence is *N*, which is divided into *n* action segments after the action segmentation and is denoted as *N*_1_, *N*_2_,…, *N*_*n*_. Similar to the musical characteristics, the action characteristics in this section are also composed of rhythmic characteristics and intensity characteristics, and the characteristics of the action *N*_*i*_(1 ≤ *i* ≤ *n*) fragment are

(19) $$\begin{array}{c} \text{motion feature }\left(f\right)=\left[\begin{array}{c} F_{R}^{\text{Motion}}\left(f\right)\\ F_{l}^{\text{Motion}}\left(f\right) \end{array}\right],\;f\in N_{i}, \end{array}$$

where *f* is the frame number of the action clip and *F*_*R*_^Motion^ and *F*_1_^Motion^ are the rhythm and intensity characteristics *N*_*i*_ of the action clip *N*_*i*_, respectively.

The local minimum of the *W*(*f*) sum of the displacement differences of the joints in two adjacent frames corresponds to the possible action rhythm:

(20) $$\begin{array}{c} W\left(f\right)=\sum_{k=1}^{c}\alpha^{\left(k\right)}\cdot \left\|x_{f+1}^{\left(k\right)}-x_{f}^{\left(k\right)}\right\|, \end{array}$$

where *x* denotes the action vector, *x*_*f*_^(*k*)^ denotes the *k*th dimensional action data of the first *f* frame, and *c* is the vector dimension of each frame of action. Since each joint point has a different range of movable motion and different contributions and importance to the action rhythm feature, weights *α*^(*k*)^ are introduced to weight the skeletal displacement.

In summary, the rhythmic characteristics of the *N*_*i*_ action fragment defined in this paper are

(21) $$\begin{array}{c} F_{R}^{\text{Motion}}\left(f\right)=\left\{\begin{array}{cc} 1, & f\text{ is the beat moment,}\\ 0, & \text{else,} \end{array}\right.,\;f\in M_{i}. \end{array}$$

The movement intensity characteristic is the average of the intensity of each frame in the same rhythm cycle, i.e.,

(22) $$\begin{array}{c} F_{l}^{\text{Motion}}\left(f\right)=\sum_{i=f_{R}^{s}}^{f_{R}^{e}}\frac{W\left(i\right)}{f_{R}^{e}-f_{R}^{s}+1}. \end{array}$$

In order to make full use of the action data and obtain a better matching effect, a certain proportion of scaling is allowed in matching and the scaling proportion used in this paper is from 0.9 to 1.1 for all numbers in the range of step size 0.05. The *M*_*i*_ formula for calculating the rhythm matching degree of *N*_*i*_ is

(23) $$\begin{array}{c} \hat{s}=\max_{s,f_{0}}\sum_{f=1}^{L_{\text{music}}}\frac{F_{R}^{\text{Music}}\left(f\right)\cdot F_{R}^{\text{Motion}}\left(s\cdot f+f_{0}\right)}{F_{R}^{\text{Music}}\left(f\right)+F_{R}^{\text{Motion}}\left(s\cdot f+f_{0}\right)},\;f_{0}\in \left[0,\;L_{\text{motion}}-s\cdot L_{\text{music}}\right],\;s\in \left[0.9,1.1\right]. \end{array}$$

where *L*_music_ and *L*_motion_ are the lengths of *M*_*i*_ and *N*_*i*_, respectively, *s* is the scaling factor, and *f*_0_ is the translation.

Based on the matching result, the *t* action segments with the most matching rhythm are selected for each music segment, which is denoted as *N*_*i*,1_, *N*_*i*,2_,…, *N*_*i*,*t*_,  *N*_*i*,*j*_ ∈ *N*, 1 ≤ *i* ≤ *m*, 1 ≤ *j* ≤ *t*_0_.

The intensity matching formula for the music clip *M*_*i*_ and the action clip *N*_*i*_ is

(24) $$\begin{array}{c} \hat{D}=\sum_{f=1}^{L_{\text{music}}}\sqrt{\frac{F_{1}^{\text{Music}}\left(f\right)}{\sum_{k=1}^{L_{\text{music}}}F_{1}^{\text{Music}}\left(k\right)}\cdot \frac{F_{1}^{\text{Motion}}\left(f\right)}{\sum_{k=1}^{L_{\text{motion}}}F_{1}^{\text{Motion}}\left(k\right)}}, \end{array}$$

where *L*_music_ is the length of *M*_*i*_ and *L*_motion_ is the length of *N*_*i*_.

### 2.4. Choreography and Synthesis

In this paper, we use the interpolation algorithm of intermediate frames to interpolate between the end *k* frames of action clip *M* and the intermediate action of action clip *N* according to the interpolation weights to get the final interpolated action. In order to avoid that the interpolation action lasts too long and affects the perception, the value of *k* cannot be too large and *k* = 14 is taken in this paper. The schematic diagram of intermediate frame interpolation process is shown in Figure 5.

Let the length of action fragment *M* be *m*, the last *k* frames of action are denoted as *M*_*m*−*k*+1,…,*m*_={*f*_*m*−*k*+1_^*M*^, *f*_*m*−*k*+2_^*M*^,…, *f*_*m*_^*M*^}, and the first *k* frames of intermediate action of action fragment *N* are denoted as *N*_1,…,*k*_={*f*_1_^*N*^, *f*_2_^*N*^,…, *f*_*k*_^*N*^}; firstly, the starting position of *N*_1,…,*k*_ intermediate action is translated to *M*_*m*−*k*+1_, andinterpolation action is synthesized *P*_1,…,*k*_, where *P*_1,…,*k*_={*f*_1_^*P*^, *f*_2_^*p*^,…, *f*_*k*_^*P*^}. The linear interpolation of node displacement is performed:

(25) $$\begin{array}{c} p_{i}^{p,s}=\alpha \left(i\right)f_{m-k+i}^{M,s}+\left(1-\alpha \left(i\right)\right)f_{i}^{N,s},\;1\leq i\leq k,\\ \alpha \left(i\right)=2\cdot {\left(\frac{i}{k}\right)}^{3}-3\cdot {\left(\frac{i}{k}\right)}^{2}+1,\;0\leq i\leq k-1, \end{array}$$

where *p*_*i*_^*P*,*s*^ represents the coordinate of the *s*-th node of the *i*-th frame of the *P* action clip and *α*(*i*) is the interpolation weight.

## 3. Experiments and Results

Based on mixed density network (MDN), the effectiveness of multilevel music and action feature matching algorithm and the effect of comprehensive dance are experimentally evaluated.  Figure 6 shows the pose snapshot of the synthesized dance. From the intuitive visual effect, the choreography algorithm of this paper can be considered effective. Firstly, the overall characteristics of “Tokyo Teddy Bear” are extracted, the BPM value is calculated to be 126.05 and the change note duration is 1.93, and the candidate movement database is chosen to be generated using the fast house dance movement generation model. Observing the final dance effect, we can feel that the dance matches the rhythm and intensity of the target music to some extent and the movements are smooth and coherent.

As shown in Figure 7, the skeletal motion speed features of both arms are extracted in this paper and the effect of the feature extraction algorithm is evaluated by the visual effect of the motion segments. By observation, the arm movements in the fifth segment do change faster than those in the seventh segment, indicating *v*_*i*_^Arm^ such that the numerical values can accurately reflect the arm movement speed, so the local skeletal velocity feature extraction algorithm proposed in this paper is effective.

As shown in Figure 6, this paper verifies the effectiveness of the dance spatiality feature extraction algorithm by comparing the spatiality metric *e*_*i*_ of the action clips with the real root node motion trajectory. The spatiality of the first action fragment (frames 1–13) is weak, and the spatiality of the second action fragment (frames 14–24) is strong, as judged by the values of *e*_*i*_.

In order to verify whether the judgment is accurate, the motion paths of the root nodes of the two action fragments projected on the ground are drawn separately, as shown in Figure 8, where the blue path corresponds to the first action fragment and the red path corresponds to the second action fragment. After observation, it can be found that the range of motion trajectory of the second action fragment is indeed larger, which indicates that the above judgment is accurate and the action fragment can be described spatially by the spatiality metric of the action fragment, so the spatiality feature extraction algorithm proposed in this paper is effective.

## 4. Summary and Outlook

Based on the mixed density network (MDN), this paper generates the dance matching with the target music through three steps, motion generation, motion screening, and feature matching, and implements a music arrangement algorithm based on the mixed density network, which can generate the dance matching with the target music. This paper proposes a multilevel music and action feature matching algorithm, which combines global feature matching with local feature matching, in order to improve the unity and integrity of music and action. The experimental results show that after adding the control based on the overall music characteristics, the speed and other characteristics of each action segment in the final synthesis result are more consistent and the overall arrangement is more beautiful. Compared with the original motion data, the motion data generated by the mean method is more real and the consistency of the filtered motion data is significantly improved. Compared with the existing music arrangement algorithms, the algorithm proposed in this paper improves the consistency and novelty of movement, the compatibility with music, and the controllability of dance characteristics. Therefore, the algorithm in this paper is technically changing the way of artistic creation, which provides the possibility for the development of motion capture technology and artificial intelligence. The algorithm improves the unity and coherence of music and action. However, other problems in the application of neural network in image and sound signal analysis still need further research.

## Figures and Tables

**Figure 1:** Schematic diagram of the overall structure of the motion generation model.

**Figure 2:** Network structure of the action generation model.

**Figure 3:** Model loss: training set.

**Figure 4:** Model loss: validation set.

**Figure 5:** Schematic diagram of the interpolation process of the intermediate frames.

**Figure 6:** Spatiality metric of action fragments.

**Figure 7:** Average arm speed of the action segment.

**Figure 8:** Root node motion path.

**Table 1:** Parsing the VMD file bone keyframe data block to obtain part of the data.

	Frame number	Bone ID	Bone displacement			Number of skeletal rotation pions			
	0	1	2	3	4	5	6	7	8
0	0.000	0.000	0.066	0.000	5.970	0.000	0.379	0.000	−0.925
1	0.000	1.000	0.000	0.000	0.000	0.000	0.000	0.000	1.000
2	0.000	2.000	0.000	0.000	0.000	−0.257	0.000	0.000	0.966
3	0.000	3.000	0.000	0.000	0.000	−0.125	0.000	0.000	0.000
4	0.000	4.000	0.000	0.000	0.000	0.000	0.000	−0.105	0.995

**Table 2:** Details of the various types of data in the dataset.

Dance style	Information				
	Overall speed	Number of clips	Frame speed	Frame rate	Duration (min)
House dance	Quick	54	Quick	285393	158.6
			Slow	26428	14.7
	Slow	35	Quick	157175	87.3
			Slow	54034	30.0

Street dance	Quick	67	Quick	357287	198.5
			Slow	18159	10.1
	Slow	6	Quick	26615	14.8
			Slow	9074	5.0

Modern dance	Quick	5	Quick	22780	12.7
			Slow	252	0.1
	Slow	25	Quick	42627	23.7
			Slow	57521	32.0

## Data Availability

The data used to support the findings of this study are available from the corresponding author upon request.
